RETRACTED

# The Effectiveness of Pictorial Aesthetics Based on Multiview Parallel Neural Networks in Art-Oriented Teaching

**DOI:** 10.1155/2021/3735104

**Published:** 2021-08-23

**Authors:** Liang Gang, Gao Weishang

**Affiliations:** ^1^College of Art and Design, Taizhou University, Taizhou 318000, Zhejiang, China; ^2^School of Electronics and Information Engineering, Taizhou University, Taizhou 318000, Zhejiang, China

## Abstract

How to effectively improve the effectiveness of art teaching has always been one of the hot topics concerned by all sectors of society. Especially, in art teaching, situational interaction helps improve the atmosphere of art class. However, there are few attempts to quantitatively evaluate the aesthetics of ink painting. Ink painting expresses images through ink tone and stroke changes, which is significantly different from photos and paintings in visual characteristics, semantic characteristics, and aesthetic standards. For this reason, this study proposes an adaptive computational aesthetic evaluation framework for ink painting based on situational interaction using deep learning techniques. The framework extracts global and local images as multiple input according to the aesthetic criteria of ink painting and designs a model named MVPD-CNN to extract deep aesthetic features; finally, an adaptive deep aesthetic evaluation model is constructed. The experimental results demonstrate that our model has higher aesthetic evaluation performance compared with baseline, and the extracted deep aesthetic features are significantly better than the traditional manual design features, and its adaptive evaluation results reach a Pearson height of 0.823 compared with the manual aesthetic. In addition, art classroom simulation and interference experiments show that our model is highly resistant to interference and more sensitive to the three painting elements of composition, ink color, and texture in specific compositions.

## 1. Introduction

Currently, the large teacher-student ratio in college art classrooms, the existence of strong interaction, i.e., between individual teachers and groups of students, and the high frequency of drawing exams have led to problems in art teaching and art classrooms [1]. The difficulty of drawing exams is not conducive to the development of the art classroom with the main purpose of improving students' drawing quality. The pursuit of teaching effectiveness is the essence of teaching, and learning is also the essence of teaching curriculum reform, which is the inevitable requirement to achieve the connotation development of education. However, in the contemporary school teaching practice, there are still problems that teachers try to teach, students do not learn, and the quality of teaching is mediocre [2, 3]. Therefore, improving the effectiveness of classroom teaching has become one of the core topics of the current curriculum and teaching reform, and the study of effective classroom teaching strategies is a key factor in addressing this challenge. After continuous exploration and research, the authors learned that effective teaching theory has been extensively used in the teaching of various subjects and has achieved significance results [4], and an efficient and effective teaching mode has taken shape. In view of this, it is also imperative to promote the effectiveness of art teaching.

RETRACTED

There are many problems in art classrooms; for example, art teachers are relatively weak in many countries, making it difficult to develop later more specialized art curriculum training programs, and schools lack attention to this aspect of curriculum application [5]. At the same time, art teachers need to manage a large number of students at the same time and are unable to detect whether each student completes the exercise in a quality and quantity manner. For example, in a semester-long art study course in a university, teachers lead students in drawing exercises, and under normal circumstances, students fail to memorize and draw accurately, and the subsequent lack of attention makes their own course projects limited [6]. Students will rush to study at the end of the actual test period, which results in nonstandardized drawing, or even the drawing content is done roughly [7]. In addition, some college art classes lack effective teaching methods to enhance students' drawing ability. In general, four-year majors usually set up two years of art classes. During this period, students' drawing ability is low and even fails to meet the drawing test standard, because they do not form good drawing habits [8, 9].

Traditional art training programs are too boring and cannot stimulate students' interest. For example, ink painting is a typical representative of traditional Chinese painting art, which creates a hierarchy of dry and wet ink colors through ink and water tone and brushwork changes, such as colorful artistic effects and high aesthetic value [10]. The traditional aesthetic assessment of ink painting can only be described qualitatively by connoisseurs, and the results are subjective and uncertain. In addition, the number of ink painting images stored on the Internet is just so large that it is impractical to invite a small number of highly qualified experts to evaluate them one by one manually. If they can be quantitatively evaluated by computer in an efficient and automatic way, it will help beginners to evaluate the aesthetics of their works in the process of learning ink painting, which is of great significance for teaching ink painting and also has promising applications in the fields of advanced ink painting retrieval and recommended display of digital Chinese painting art galleries [11]. With the help of deep learning, it is possible to realize the performance of students' paintings based on situational interaction, such as the relatively boring ink painting, and guide students' interest in painting through deep learning evaluation mechanism.

RETRACTED

Computational aesthetics, on the other hand, are a research direction that has emerged only in recent years, even though computers can simulate the human visual system and aesthetic thinking and automatically make feasible aesthetic decisions in relevant applications. Most of this current work has been done with photographs and Western paintings as research objects, based on image aesthetic evaluation datasets [12, 13], or manually designed visual features [13], and in recent years using deep convolutional neural networks to automatically extract high-level aesthetic features [14], while the latter have achieved superior performance in aesthetic classification and evaluation tasks, but they cannot be fully applied to quantitative aesthetic ink painting in the quantitative assessment of ink painting. Moreover, the aesthetic properties of ink paintings of the same subject matter vary according to their content, making it difficult to apply a single aesthetic model to all subject matter types. Most of the existing methods train independent aesthetic models based on specific types of scenes or a priori knowledge, which have certain scenario limitations [15].

In order to address the above challenge, this study proposes an aesthetic adaptive quantitative assessment method based on deep learning, taking traditional ink painting as the research object in art teaching and combining it with art professional appreciative theory. MVPD-CNN is designed to extract deep aesthetic features based on the aesthetic characteristics of ink painting and adaptive image blocks as multiple inputs, so as to better capture and quantify the aesthetic perception information of ink color, brush strokes, and composition of different subjects in ink painting [16]. We also construct an adaptive depth aesthetic evaluation model for ink painting based on the subject matter content query mechanism.

Furthermore, in response to the current situation of low effectiveness of art teaching in universities, the use of deep learning to assist art teaching is proposed. First, the connotation and meaning of art teaching effectiveness are analyzed. The experimental results demonstrate that the aesthetic evaluation of art teaching based on artificial intelligence can significantly improve students' drawing ability, endurance, and sensitivity. The application of artificial intelligence in college art teaching realizes the diversification and multifunctionality of college art teaching management methods, which are important for establishing a new teaching method that is truly suitable for modern art teaching.

RETRACTED

## 2. Related Work

### 2.1. Hardware Supports in Art Teaching

Traditional electronic devices such as video recorders and projectors are the most common electronic means used in modern education, and these devices are also used in art education [17]. For example, teachers can make art knowledge more vivid through pictures and videos. In music education, for example, with the help of traditional electronic devices, students can learn knowledge more systematically and faster [18]. This type of education can increase learners' interest, teach more content in a certain amount of time, and improve teachers' work efficiency. The purpose of exploring the application of AI in art teaching is to present art knowledge to students in a more intuitive way, create a better learning atmosphere, showcase design works that combine art and technology, help students enter the world of artists' creations, allow students to truly immerse themselves in the masterpieces of great artists, break the limitations of time and place, and allow viewers to observe the details of art works in a more intuitive way [19–21]. However, due to the lack of AI hardware facilities in art teaching, it is difficult to achieve the expected art teaching effect or teaching goal.

### 2.2. Software Support in Art Teaching

The current commonly used computer-assisted instruction (CAI) makes comprehensive use of multimedia, hypertext, artificial intelligence, network communication, knowledge base, and other computer technologies to overcome the shortcomings of traditional art teaching in a single, one-sided teaching context [9, 22, 23]. It can effectively shorten the learning time of art education, improve the quality and efficiency of teaching, and achieve the most optimal teaching objectives. For example, there are adaptive learning systems for university teachers and students; there are teaching materials that can interact with students and change course content based on their answers to random tests; there are intelligent teaching materials customized to students' individual needs; and there are cases where the interface is more appropriately designed based on image analysis to improve user experience, etc. [6, 24, 25]. Although traditional CAI improves students' learning efficiency and motivation to a certain extent, however, it does not fully understand the students' learning situation, cannot be customized, and cannot guarantee that every student can actively participate in teaching. Therefore, if we want students to participate more actively in the teaching process, if we want to collect the learning situation of individual students and give different instructions through human-computer interaction, then we should combine multimedia technology with technical breakthroughs in artificial intelligence to provide more powerful technical support for modern teaching [26].

RETRACTED

### 2.3. Art Teaching Modes

At present, the AI-based art teaching mode in colleges and universities is mainly to teach art teaching content with the help of Internet technology and online platforms [27]. In this process, various educational applications and online education websites have emerged, such as massive open online courses (MOOC), microlecture online video, flipped classroom, PAD classroom, and Tencent classroom [14, 28, 29]. This teaching mode innovates the interactive cognitive process of teaching and supports a variety of functions such as play, stop, and slow play, which enables students to make use of scattered time for learning and effectively control the learning speed [30]; at the same time, it breaks through the limitation of location, effectively solves the drawbacks of the traditional offline teaching mode, and greatly improves the utilization rate of teachers [31]. However, this art teaching model ignores the experiential and holistic nature emphasized in art teaching, and especially in the case of a large number of students, art teachers and students can only teach and learn art knowledge in a one-to-one format, which cannot provide students with an art teaching atmosphere [32]. In addition, because artificial intelligence technology is not mature enough, the art teaching model based on artificial intelligence can no longer meet the requirements of intelligent teaching, resulting in a disconnection between modern art teaching concepts and intelligent teaching mode.

### 2.4. AI for Art Classrooms Construction

Artificial intelligence (AI) technology can automatically perform data processing [8, 33]. Processing and judging data are derived from outside sources. AI relies on computer systems, machine learning, psychology, etc. Currently. There are a lot of discussions about introducing some AI applications in college art classrooms, among which Apple is one of the many applications. The construction and reform of these systems in college classrooms mainly focus on improving students' interest in learning, the reform of art teaching content is relatively simple, and the emergence of these teaching methods is basically aimed at students, which is not conducive to improving teachers' teaching efficiency [11, 28]. Based on the above, this paper improves the existing classroom on the basis of Figure 1 and proposes a more reliable, efficient, and easy-to-operate computer-aided teaching system, which can be applied to athletics, long jump, and other art venues, consisting of AI computer system, human-machine interface, etc., management terminal display equipment, venue sensing equipment, venue prompting equipment, and wireless sensing prompting equipment, as shown in Figure 1.

RETRACTED

AI art teaching completely overturns the traditional teaching model, mainly changing the structure of educational resources, teaching feedback, and evaluation mechanisms into an intelligent teaching method [34]. Through AI platform, teachers and learners are accurately connected to form a new multilevel, wide-area and multifaceted AI art teaching system. Educational resources and teaching are mostly built on a digital basis, with more emphasis on the diversity and reoptimization of resources. What is worth our attention is that AI art teaching is built on top of numerous AI devices and big data processing centers. It cannot be separated from technical support and environment construction, but the teaching service it provides is intelligent, novel, smart, and advanced [35].

## 3. MVPD-CNN

### 3.1. Network Infrastructure

In this study, the aesthetic scoring task of ink painting is represented as a regression modeling problem for predicting continuous scores. The ink painting input image is represented as *x*_*n*_, and a deep CNN complex is constructed to automatically learn the regression mapping function *f* : *ℜ*^2^⟶*ℜ* to predict the aesthetic score ${\hat{y}}_{n}=f\left(x_{n}\right)$. Given the ink painting training sample {(**x**_*n*_, *y*_*n*_)}_*n*∈(1, *N*)_, where N is the training set size, *y*_*n*_ is the artificial benchmark score, and W is the set of network model parameters. The entire network is optimized by minimizing the Euclidean regression loss function.

(1) $$\begin{array}{c} l\left(W\right)=\frac{1}{2N}\sum_{n=1}^{N}{\left\|{\hat{y}}_{n}-y_{n}\right\|}_{2}^{2}+\lambda {\left\|W\right\|}_{2}^{2}, \end{array}$$

where *λ*‖**W**‖_2_^2^ denotes the weight decay regularization; *λ* denotes the regular strength coefficient. In order to overcome the overfitting problem of the smaller ink painting dataset, the pretrained model of VGG16 [10, 36] on ImageNet [17, 37] is used as the baseline network for migration learning, as shown in Figure 2 and the network structure consists of 13 convolutional layers and 3 fully connected layers, fixing the structure of the first 12 convolutional layers, while adjusting the other layers as follows.

  Step 1: A subject matter convolutional layer is designed to replace layer 13 of the original network. The subject matter layer consists of six parallel groups of convolutional networks (64 convolutional kernels each), which are used to extract the aesthetic descriptors of six different subjects in ink painting: flowers, birds, grasses and insects, shrimps and crabs, fruits and vegetables, animals, landscapes, and people. The output of this layer is connected to the first fully connected layer through averaging pooling, which enables the network to have a robust adaptive learning capability for different ink painting themes.
  Step 2: Replace the 1000-dimensional classification probability of the last fully connected layer with a regression layer containing 1 neuron to predict the beautiful score, and replace the softmax loss layer with a Euclidean loss layer for the final output.
  Step 3: The number of neurons in the first two fully connected layers is reduced from 4096 to 512 and 256, thus reducing the number of parameters, preventing overfitting, and facilitating feature cascading. After the modification, the entire network infrastructure is shown in Table 1.

RETRACTED

In order to extract aesthetic features more effectively according to different ink painting topics, a pretraining method is designed to initialize the model. In the initialization stage of the network parameters, the pretrained weights of the first two convolutional layers of the VGG16 model are fixed as the initialization parameters of the corresponding layers in the network, while, for the 13th convolutional layer, each convolutional group is fine-tuned individually using the training data of the corresponding subject matter, and the corresponding network weights are updated [15]. When all groups are trained, each group of training weight is initialized by linking them to the ink painting topic convolutional layer in parallel, thus ensuring that each topic category has its own corresponding neuron activation. The remaining two fully connected layers and the regression layer parameters are initialized randomly.

## 4. Multiview Parallel Deep CNN

The aesthetic perception of ink painting needs to consider the overall and local perspectives; for example, landscape painting focuses on the “five character method” and “far method” in the overall composition, while there is the distribution of white space and sparse contrast in the local area [12, 22]. In this paper, we design a deep CNN architecture with multiple viewpoints in parallel, as shown in Figure 3. The global images of different expressions are first extracted according to the aesthetic criteria and basic structure of ink painting, and the image blocks are adaptively selected as multiple inputs; then each input is merged with the features extracted by the respective VGG16 networks through the statistical aggregation structure; finally, the global and local features of the output are cascaded to perform aesthetic prediction.

RETRACTED

Specifically, the model we designed is shown in Figure 3: firstly, the input, which is simultaneously input in two modules, the global view for image query, and the local view for feature adaptive selection; in the global view module, module representation, storage representation, and composition representation are operated separately and then input into the respective corresponding VGG16; similarly, the local view module inputs the adaptively selected *p* from the image. Similarly, the adaptively selected *p* from the image is input into the corresponding VGG16 in the local view module, and then the outputs of VGG16 of each channel in the global and local modules are stitched together, and then these VGG16 stitches are statistically aggregated, and then the depth features are mined for the prediction of the overall model.

### 4.1. Ink Painting Global and Local View Input

For the global view input, in ink color, ink painting is expressed through the contrast between colored ink strokes and white space, and the change of intensity and shade of gray. Here, the original ink painting, the H and S channels of HSV map [7], and the grayscale map are selected as the input; for the brush strokes, the wavelet coefficients of the image contain rich edge energy information, which can capture the information of local details of ink painting strokes and the texture characteristics of typical brush strokes. In this paper, the wavelet coefficient matrix of Daubechies layer 1 is used as texture input, and for the composition, the spatial distribution structure of each element in the image is analyzed by calculating the saliency map of the ink painting, and the original image is segmented into several uniform regions using the SLIC [14, 29] super-pixel segmentation method 1 as shown in Figure 4(a), followed by the histogram comparison-based method proposed by [29]. to calculate the grayscale saliency map as shown in Figure 4(b), the higher the significance value of the brighter region is, the more important it is in terms of aesthetic vision.

For the local view input, the ink painting is represented as a collection of cropped image blocks, where *M* denotes the number of image blocks. Different from the random cropping method, this paper adopts an adaptive strategy to extract the image blocks with the most aesthetic perceptual information in the ink painting, with the following criteria: saliency detection can highlight the visually important regions in the picture, so the saliency map is used to select the most recognizable and informative regions in the image; the important aesthetic details in the ink painting are expressed through the relationship between different subjects and the background, so that the pattern diversity within the image blocks is ensured; the spatial distance between different image blocks is constrained, so that the overlap between the image blocks is as small as possible. Therefore, the ink painting image block selection is considered as an optimization problem, and the objective function is defined.

(2) $$\begin{array}{c} \left\{c^{*}\right\}=\arg\max F\left(S,D_{p},D_{s}\right),\\ F\left(.\right)=\sum_{i=1}^{M}S_{i}+\sum_{i\neq j}^{M}D_{p}\left(N_{i},N_{j}\right)+\sum_{i\neq j}^{M}D_{s}\left(c_{i},c_{j}\right), \end{array}$$

where {*c*_*m*_^*∗*^}_*m*∈[1, *M*]_ denotes the coordinates of each center of the optimal image block set, *S*_*i*_ denotes the normalized significance value of each image block *p*_*i*_, and *D*_*p*_(.) and *D*_*s*_(.) denote the pattern distance function and the Euclidean spatial distance function, respectively. In this paper, a multivariate Gaussian is used to model each image block *p*_*m*_ pattern, i.e.,

(3) $$\begin{array}{c} N_{m}={\left\{{\left\{N_{e}\left(\mu_{e},\Sigma_{e}\right)\right\}}_{m},{\left\{N_{c}\left(\mu_{c},\Sigma_{c}\right)\right\}}_{m}\right\}}_{m\in \left[1,M\right]}, \end{array}$$

where {*N*_*e*_(*μ*_*e*_, Σ_*e*_)}_*m*_ and {*N*_*c*_(*μ*_*c*_, Σ_*c*_)}_*m*_ represent the stroke edge distribution and shade chroma distribution of the image block, respectively, and the mode distance is used to measure the difference between the two image blocks.  Figure 5 shows the results of several image blocks extracted with the adaptive selection strategy, all of which are 224 *∗* 224 *∗* 3. This method not only effectively selects the most prominent regions (e.g., flowers, loquats, and birds), but also captures the pattern diversity between the subjects of different ink paintings and the left-white background (e.g., tree trunks and landscapes, branches and leaves and grass, and insects).

RETRACTED

### 4.2. Statistical Aggregation Structure

The statistical aggregation structure is used to combine the features of each path through the output of VGG16 network. Taking the local image blocks as an example, the set of image block features output by the VGG16 network group is represented by **D**={**d**_*m*_}_*m*∈[1, *M*]_, where **d**_*m*_ is a k-dimensional vector, *T*_*m*_={**d**_*mk*_}_*m*∈[1, *M*]_ is used to represent the set of all kth components, and ⊕ is used to represent the vector cascade operation. The statistical layer consists of a statistical function *F*_Agg_={*F*_Agg_^*u*^}_*u*∈[1, *U*]_, and the output cascade *U*={*F*_min_, *F*_max_} of this set is aggregated by the fully connected layer to produce a *k*_stat_-dimensional feature vector. The whole structure function is expressed as

(4) $$\begin{array}{c} g\left(D\right)=W\times \left({⊕}_{u=1}^{U}{⊕}_{k=1}^{K}F_{\text{Agg}}^{u}\left(T_{k}\right)\right), \end{array}$$

where **W** ∈ *ℜ*^*K*_stat _×UK^ is the fully connected layer parameter, and the statistical aggregation structure of *M*=4, *K*=3 is shown in Figure 6, and *M*=5, *K*=256 is set in the experiment.

## 5. Application Performance Analysis of AI in Art Teaching

To measure the effectiveness of the application of AI in modern art teaching, the effect of its application must be analyzed. Guided by the principles of science, objectivity, and relevance, this study, through expert consultation, selects several indicators such as art teaching mode, art teaching method, art teaching content, art classroom teaching atmosphere, art teaching means, and art teaching effect to analyze the application performance of AI in art teaching and constructs the weight judgment matrix of performance indicator through expert scoring method as follows:

(5) $$\begin{array}{c} A=\left[\begin{array}{ccccccc} 1 & 1 & 1 & 1 & 1 & 1 & 2\\ 1 & 1 & 2 & \frac{1}{3} & \frac{1}{3} & \frac{1}{2} & \frac{1}{2}\\ 1 & \frac{1}{2} & 1 & 1 & \frac{1}{2} & \frac{1}{3} & \frac{1}{3}\\ 1 & 3 & 2 & 1 & \frac{1}{3} & \frac{1}{3} & \frac{1}{2}\\ 1 & 3 & 2 & 3 & 1 & \frac{1}{3} & 3\\ 1 & 2 & 3 & 3 & 3 & 1 & 3\\ \frac{1}{2} & 2 & 3 & 2 & \frac{1}{3} & \frac{1}{3} & 1 \end{array}\right]. \end{array}$$

Using the AHP method [7, 18, 22], the sequence of weights *W* corresponding to the above performance indicators was derived as

(6) $$\begin{array}{c} W=\left\{0.144,0.088,0.077,0.103,0.196,0.268,0.124\right\}. \end{array}$$

For a given performance analysis object *P*, its initial value relative to performance indicator *j* is *v*_*j*_(*P*), and if the indicator is positive, its value, after normalization, is *u*_*j*_(*P*).

(7) $$\begin{array}{c} u_{j}\left(P\right)=\frac{v_{j}\left(P\right)-v_{j}^{\min}\left(O\right)}{v_{j}^{\max}\left(O\right)-v_{j}^{\min}\left(O\right)}, \end{array}$$

where *v*_*j*_^min^(*O*) is the maximum value of indicator *j* of *P* object and *v*_*j*_^min^(*O*) is the minimum value of indicator *j* of *P* object.

(8) $$\begin{array}{c} u_{j}\left(P\right)=\frac{v_{j}^{\max}\left(O\right)-v_{j}\left(P\right)}{v_{j}^{\max}\left(O\right)-v_{j}^{\min}\left(O\right)}, \end{array}$$

After expert consultation, the performance of the application of AI in modern art teaching is divided into *M* levels, and the gray clustering function of the performance indicator *j* on the degree of performance of the application of the *k*-th level is *ϕ*_*j*_^*k*^(*u*)=*ϕ*_*j*_^*k*^[*u*_*j*_^*k*^(*a*), *u*_*j*_^*k*^(*b*), *u*_*j*_^*k*^(*c*), *u*_*j*_^*k*^(*d*)], where *u*_*j*_^*k*^(*a*), *u*_*j*_^*k*^(*b*), *u*_*j*_^*k*^(*c*), *u*_*j*_^*k*^(*d*) is the turning point of *ϕ*_*j*_^*k*^(*u*), namely,

(9) $$\begin{array}{c} \phi_{j}^{k}\left(u\right)=\left\{\begin{array}{cc} 0, & u\notin \left[u_{j}^{k}\left(a\right),u_{j}^{k}\left(d\right)\right],\\ 1, & u\in \left[u_{j}^{k}\left(b\right),u_{j}^{k}\left(c\right)\right],\\ \frac{u-u_{j}^{k}\left(a\right)}{u_{j}^{k}\left(b\right)-u_{j}^{k}\left(a\right)}, & u\in \left[u_{j}^{k}\left(a\right),u_{j}^{k}\left(b\right)\right],\\ \frac{u_{j}^{k}\left(d\right)-u}{u_{j}^{k}\left(d\right)-u_{j}^{k}\left(c\right)}, & u\in \left[u_{j}^{k}\left(c\right),u_{j}^{k}\left(d\right)\right]. \end{array}\right. \end{array}$$

In particular, if *u*_*j*_^*k*^(*a*)=*u*_*j*_^*k*^(*d*), then *ϕ*_*j*_^*k*^(*u*) is the gray clustering function for the lower bound metric, i.e.,

(10) $$\begin{array}{c} \phi_{j}^{k}\left(u\right)=\left\{\begin{array}{cc} 1, & u\in \left[0,u_{j}^{k}\left(c\right)\right],\\ \frac{u_{j}^{k}\left(d\right)-u}{u_{j}^{k}\left(d\right)-u_{j}^{k}\left(c\right)}, & u\in \left[u_{j}^{k}\left(c\right),u_{j}^{k}\left(d\right)\right],\\ 0, & u\in \left[u_{j}^{k}\left(d\right),1\right]. \end{array}\right. \end{array}$$

If *u*_*j*_^*k*^(*b*)=*u*_*j*_^*k*^(*c*), then *ϕ*_*j*_^*k*^(*u*) is a gray clustering function of medium measure, i.e.,

(11) $$\begin{array}{c} \phi_{j}^{k}\left(u\right)=\left\{\begin{array}{cc} 0, & u\in \left[0,u_{j}^{s}\left(a\right)\right],\\ \frac{u-u_{j}^{s}\left(a\right)}{u_{j}^{s}\left(b\right)-u_{j}^{s}\left(a\right)}, & u\in \left[u_{j}^{s}\left(a\right),u_{j}^{s}\left(b\right)\right]\\ \frac{u_{j}^{s}\left(c\right)-u}{u_{j}^{s}\left(c\right)-u_{j}^{s}\left(b\right)}, & u\in \left[u_{j}^{s}\left(b\right),u_{j}^{s}\left(c\right)\right],\\ 0, & u\in \left[u_{j}^{s}\left(c\right),1\right]. \end{array}\right. \end{array}$$

If *u*_*j*_^*k*^(*c*)=*u*_*j*_^*k*^(*d*), then *ϕ*_*j*_^*k*^(*u*) is the gray clustering function for the upper limit measure, i.e.,

(12) $$\begin{array}{c} \phi_{j}^{k}\left(u\right)=\left\{\begin{array}{cc} 1, & u\in \left[u_{j}^{k}\left(b\right),1\right],\\ \frac{u-u_{j}^{k}\left(a\right)}{u_{j}^{k}\left(b\right)-u_{j}^{k}\left(a\right)}, & u\in \left[u_{j}^{k}\left(a\right),u_{j}^{k}\left(b\right)\right],\\ 0, & u\in \left[0,u_{j}^{k}\left(a\right)\right]. \end{array}\right. \end{array}$$

Then, for *P* objects, the weighted gray correlation *ξ*^*k*^(*u*) of each indicator to the *k*th performance degree is

(13) $$\begin{array}{c} \xi^{k}\left(u\right)=\sum_{j=1}^{n}\left(w_{j}*\phi_{j}^{k}\left(u\right)\right). \end{array}$$

If satisfied

(14) $$\begin{array}{c} \xi^{i}\left(u\right)=\max_{1\leq k\leq M}\left(\xi^{k}\left(u\right)\right),\;1\leq i,k\leq M. \end{array}$$

That is, the performance degree of *P* object is closest to the *i*th performance degree; i.e., the gray performance degree of *P* object is *i*.

RETRACTED

## 6. Experimental Results

### 6.1. Art Classroom Simulation Experiment and Analysis of Results

First, the PGPE method of the situational interaction scheme for the art classroom of MVPD-CNN is illustrated with the result graph. The state space is a one-dimensional continuous space with the initial state obeying the standard normal distribution, and the action space is also a 1-dimensional continuous space [19]:

(15) $$\begin{array}{c} s_{t+1}=s_{t}+a_{t}+\varepsilon , \end{array}$$

where *ε*⇔*N*(0, 0.3^2^) is the noise. *N*(*μ*, *σ*^2^) is used to define the Gaussian distribution. Finally, the reward function is defined as

(16) $$\begin{array}{c} R=\exp\left(-\frac{s^{2}}{2}-\frac{a^{2}}{2}\right)+1. \end{array}$$

We compared four algorithms, including the proposed one:

  PGPE: our simple method according to MVPD-CNN
  PGPEOB: a PGPE method for the best baseline
  R-PGPE: a PGPE method proposed in this paper that includes only variance regularity

We first discuss how the strategy parameters change. In this section, updated trajectories with three different parameters are studied by setting different starting positions (average parameters of −1.6, −1.0, −0.4, −0.1). Also, the parameter *τ* is placed at 1, and 10 trajectory samples are collected for each strategy iteration process. As shown in Figure 7(a), it can be seen that the plain PGPE method cannot update the parameters to the maximum gain region in 20 iterations, and at least one trajectory of R-PGPE reaches the target (as shown in Figure 7(b)), thus proving the effectiveness of the variance regularization method proposed in this paper.  Figure 7(c) illustrates that PGPEOB can update the direction relatively reliably. However, there is still some instability.  Figure 7(d) shows that our method gets the best performance among the four methods.

As can be observed in Figure 8, the R-PGPEOB method proposed in this paper can control the optimization process toward a better strategy. We represent the results of each method as an average of 20 runs. In each run, the strategy parameters are iterated 50 times. In each iteration, we collect two trajectory pieces of data to estimate the gradient of the objective function. Our method performs the best among the four compared methods. As shown in Figure 8, our method can get more stable results. We introduced the learning strategy module into the ink painting rendering engine.  Figure 9 illustrates an example of digital media art creation based on virtual reality and AI. The results in Figure 8 show that our method can represent the results of real art creation well. Meanwhile, after the application of AI algorithms, the results of our method will be more realistic, and the digital media can produce art creations that are more in line with the actual results.

RETRACTED

### 6.2. Aesthetic Assessment of Art Painting

In this paper, all the network training and testing were done by TensorFlow framework [9, 23], with an initial learning rate of 0.001 and 10 times reduction every 10 rounds, with a decay rate of weight and a momentum of 0.9. In this paper, 1200 works were expanded to 2400 works by horizontal mapping changes, after which all the works were randomly divided into 5 groups of 480 sketches each; a 5-fold cross-validation method [16, 24] was used, in which 4 groups were training samples and 1 group was testing sample, and the mean value was the final result of the model after using random gradient descent method. The model was trained using the random gradient descent method, and the mean value after the second experiment was the ultimate result. For model performance evaluation, the test set was selected, and the mean Pearson correlation coefficient (Rp/Sig.) [12, 24] and mean squared error (MSE) were calculated between the predicted and manually evaluated score of the aesthetic model, where Sig. is the *p*-value, which represents the significance for hypothesis testing, and higher Rp and Sig. <0.05 mean that the model is statistically significantly correlated; and the smaller the MSE, the smaller the prediction error, and the better the model performance. This section will compare the performance of parallel deep CNN with different infrastructure and multiview input and analyze the prediction performance of the adaptive aesthetic model based on topic query.

### 6.3. Model Performance under Different Architectures and View Inputs

Firstly, we compare the aesthetic evaluation performance of single-column deep CNN networks for ink painting with different infrastructures by using the original image of ink painting as a single view input, as shown in Table 2. Among them, Arc1 denotes the original VGG16 network structure, Arc2 denotes the VGG16 network structure with only a reduced number of neurons in two fully connected layers without a topic layer, and Arc3 denotes the VGG16 network structure after modifying the 13th convolutional layer into six parallel topic convolutional groups (the base architecture used in this model). It can be seen that the model under Arc3 architecture has higher average Rp (Sig. <0.05) and lower average MSE compared with other architecture and thus has higher aesthetic evaluation performance for ink painting. This indicates that, with fewer network parameters, the network architecture and the migration learning strategy in this paper can fully utilize the general aesthetic features such as edge color in the shallow layer of the pretrained model, while combining the adaptive subject matter convolution group and the regression loss layer to effectively capture the specialized aesthetic elements of different ink painting subjects.

RETRACTED

On this basis, this section compares the prediction performance of MVPD-CNN for aesthetic perception of ink painting with different perspective inputs and compares it with the previous traditional methods, as shown in Table 3. To check and see the effectiveness of the deep learning method, the performance of MVPD-CNN with some models using manually designed features, such as AVA4 and the linear regression model proposed by [29], is compared as a benchmark. It can be seen that the aesthetic evaluation performance of all deep learning features is significantly better than the hand-designed features, thus verifying the effectiveness of deep learning for quantitative aesthetic evaluation of ink painting. This superior performance stems from the ability of deep neural networks to extract high-level aesthetic semantic features directly from the original ink paintings based on manual scoring training data.

In addition, this section also compares the MVPD-CNN model with some existing photo aesthetic evaluation models such as RAPID15, DMA-NET31, and MSDLMII, and the results are shown in Table 3. It can be seen that the MVPD-CNN model significantly outperforms the above methods in aesthetic prediction of ink paintings. The results further validate the effectiveness of the MVPD-CNN model; especially the adaptive selection strategy can effectively extract the salient areas with the most aesthetic perceptual information in ink paintings and can capture the pattern diversity between different ink painting subjects and the white background, for example, the contrast between the brush strokes and the white space formed by the contrast between solid and void, the contrast between color and ink, and the contrast between motion and stillness.

RETRACTED

Finally, this section compares the model prediction performance under different viewpoint inputs in Arc3 architecture, where SCNN-Arc3 denotes the VGG16 model that scales the original image to a fixed size of 224 *∗* 224 *∗* 3 as a single input, and MVPD-CNN-global and MVPD-CNN-local denote the parallel network models with global image and adaptive local image blocks as MVPD-CNN-global and MVPD-CNN-local represent the parallel network models with global image and adaptive local image blocks as input, respectively, while MVPD-CNN-hybrid represents the parallel network model fusing global and local view inputs. The experimental results show that the prediction performance of the three multiplexed parallel network models MVPD-CNN-global, MVPD-CNN-local, and MVPD-CNN-hybrid is better than that of the single input SCNN-Arc3 model, while the MVPD-CNN-hybrid model has a higher average Rp(sig < 0.05) and lower average MSE compared with the other single view models. The MVPD-CNN-hybrid model has a higher mean Rp(sig < 0.05) and lower mean MSE than the other single-view models and thus has a higher performance in the aesthetic assessment of ink painting. This indicates that the model is able to extract aesthetic features of ink painting from two perspectives: overall layout information and local fine details.

### 6.4. Performance Analysis of Adaptive Deep Aesthetic Model

To further validate the prediction performance of the adaptive model, the size of the adaptive subtraining set in the retrieval process was set to 50, and the depth aesthetic features extracted from the MVPD-CNN-hybrid were trained with the manual evaluation scores using SVR, and the resulting aesthetic evaluation model was denoted by IR_CNN_+SVR_DeepAesth_. The performance of this model is compared with the MVPD-CNN-hybrid as shown in Table 4. It can be seen that IR_CNN_+SVR_DeepAesth_ has higher Rp and lower MSE compared to MVPD-CNN-hybrid, and the average sig < 0.05, and Pearson's highly significant correlation between its model evaluation results and the manual aesthetic scores reached 0.823. This indicates that the adaptive model can effectively capture the influence of different subject matter content on aesthetic criteria of ink paintings, and the depth aesthetic features in the model have high predictive performance in the computational aesthetic assessment of ink paintings.

A comparison of some ink painting images that show opposing directions in terms of aesthetic perception assessment score is shown in Figure 10. Among them, the work in the top row has higher aesthetic perception scores, while those in the bottom row have lower aesthetic perception score. The values in the figure indicate that the adaptive depth aesthetic model can describe and predict the aesthetic attributes in ink paintings well and match them with human aesthetic perception. In addition, the ink painting images in the top row have more natural variations in ink intensity and shade, smoother and more orderly brush strokes, more harmonious wet and dry contrasts, and a better sense of space in the overall layout of the image compared with the bottom row. The flexible application of aesthetic criteria by different artists in different forms of expression has resulted in a very different style of ink painting. These works have large deviations from the general aesthetic guidelines of most corresponding subjects in the dataset and are easily evaluated by the model as having lower aesthetic scores, but the works of these famous masters of Chinese painting are manually evaluated as having higher aesthetic scores because of their extremely high artistic value. The abstract style of ink painting expression is the main factor that leads to a large misjudgment in the aesthetic evaluation of ink painting work, and Figure 11 shows some samples with large deviations in evaluation score.

RETRACTED

In addition, this section further compares the performance of the linear regression model based on artificial design features, the multiview parallel deep learning model MVPD-CNN-hybrid, and the adaptive deep aesthetic model based on subject query. The aesthetic prediction performance in 6 categories of ink painting subject matter is shown in Figure 12. The figure shows that IR_CNN_+SVR_DeepAesth_ significantly and consistently outperforms the other 2 models in the 6 categories, thus further demonstrating the effectiveness of the aesthetic features learned by MVPD-CNN.

### 6.5. Deep Aesthetic Model Sensitivity Analysis

To further reveal the interpretability of the deep aesthetic model, three important elements of Chinese painting, composition, ink color, and texture are experimentally interfered with here, and the sensitivity of the deep CNN response to changes in these factors is tested.

Firstly, 100 small squares with sizes ranging from 10 × 10 to 50 × 50 pixels are selected and randomly masked at any position on the ink painting image, thus interfering with the overall layout, as shown in Figure 13 corresponding to the performance results shown as blue lines in Figure 12. It can be seen that the correlation coefficient between its model prediction results and manual scoring decays rapidly with the increase of layout interference, which indicates that the deep aesthetic model is more sensitive to spatial layout.

Secondly, different grayscale coefficients *g* are set to interfere with the overall color scale of the ink painting image, and the range is from 0 to 1, and the closer to 0, the darker the image, as shown in Figure 14. It can be seen that the correlation coefficient decreases with the increase of the color scale interference as the grayscale coefficient decreases, indicating that the model is more sensitive to the change of the level of the ink grayscale.

RETRACTED

Finally, different levels of Gaussian noise are added to the ink painting image to interfere with the texture, and the larger the variance parameter *s* is, the rougher the image is, and the corresponding performance results are shown in the green line in Figure 15. It can be seen that as the variance increases, the correlation coefficient gradually decreases with the increase of noise, indicating that the depth aesthetic model is more sensitive to the brushstroke texture.

## 7. Conclusions

Effectively increasing the effectiveness of art teaching in colleges and universities has become a hot topic of utmost concern. Little work has been done on aesthetic quantitative assessment of ink painting. In this paper, we propose an adaptive computational aesthetic evaluation framework for ink painting using deep learning techniques. The framework first constructs a benchmark dataset for aesthetic evaluation of ink painting images, then extracts global and local image blocks as multiple input according to the aesthetic criteria of ink painting, and designs a multiview parallel deep convolutional neural network to extract deep aesthetic features. The experimental results demonstrate that the depth aesthetic features extracted by this model are significantly better than the traditional hand-designed features. This study not only provides a reference framework based on deep learning for computational aesthetic assessment of art, but also provides a more important reference and reference for the effectiveness of AI-based art teaching in universities.

## Figures and Tables

**Figure 1:** AI-based construction program for college art classrooms.

**Figure 2:** Deep CNN infrastructure.

**Figure 3:** MVPD-CNN.

**Figure 4:** Ink painting saliency map extraction. (a) SLIC super-pixel segmentation map. (b) Grayscale saliency map.

**Figure 5:** Example of image blocks extracted by adaptive image block selection strategy.

**Figure 6:** Statistical aggregation structure diagram.

**Figure 7:** Aggregate patterns that combine appearance and motion flow. (a) PGPE. (b) PGPEOB. (c) R-PGPE. (d) Our method.

**Figure 8:** Comparison of the average expected return of the four algorithms. (a) Digital media art creation. (b) R-PGPE. (c) Our method.

RETRACTED

**Figure 9:** Examples of digital media art creation.

**Figure 10:** Comparison of manual (blue) and model (red) assessment scores. (a) High aesthetic feeling. (b) Low aesthetic feeling.

**Figure 11:** Comparison of manual (blue) and model (red) evaluation scores for larger misclassifications.

**Figure 12:** Comparison of the aesthetic predictive performance of different ink painting subject categories.

**Figure 13:** Ink painting image under random masking of different size squares. (a) Input. (b) 10 *∗* 10 *∗* 100. (c) 20 *∗* 20 *∗* 100. (d) 30 *∗* 30 *∗* 100. (e) 40 *∗* 40 *∗* 100. (f) 50 *∗* 50 *∗* 100.

**Figure 14:** Ink painting images with different grayscale coefficients on color gradation interference. (a) Input. (b) *g*=0.9. (c) *g*=0.7. (d) *g*=0.5. (e) *g*=0.3. (f) *g*=0.1.

**Figure 15:** Variation of Pearson correlation coefficient under different interference intensities.

**Table 1:** Deep CNN infrastructure.

Number of layers	Kernel size	Feature map size
Conv1-2	3 × 3(1)	224 × 224 × 64
Max-pool l	2 × 2(2)	112 × 112 × 64
Conv3-4	3 × 3(1)	112 × 112 × 128
Max-pool 2	2 × 2(2)	56 × 56 × 128
Conv5-7	3 × 3(1)	56 × 56 × 256
Max-pool 3	2 × 2(2)	28 × 28 × 256
Conv8-10	3 × 3(1)	28 × 28 × 512
Max-pool 4	2 × 2(2)	14 × 14 × 512
Conv11-12	3 × 3(1)	14 × 14 × 512
Conv13 (6 groups)	3 × 3(1)	14 × 14 × 64
fc1		1 × 1 × 512
fc2		1 × 1 × 256
Regression		1 × 1 × 1

**Table 2:** Performance of models with different infrastructures.

Architecture	Rp/Sig	MSE
Arc 1 conv 13(512)_−_fc 4096_−_fc 4096	0.674/0.000	0.336
Arc 2 conv 13(512)_−_fc 512_−_fc 256	0.661/0.000	0.348
Arc 3 conv 13(64)_fc 512_fc 256	0.712/0.000	0.285

**Table 3:** Performance comparison between MVPD-CNN and baseline under different view inputs.

Method	Rp/Sig	MSE
AVA [16]	0.462/0.000	0.532
Zhang and Chen [23]	0.556/0.000	0.446
RAPID [13]	0.645/0.000	0.371
DMA-Net [25]	0.654/0.000	0.352
MSDLM [28]	0.669/0.000	0.344
SCNN-Arc3	0.712/0.000	0.285
MVPD-CNN-global	0.731/0.000	0.267
MVPD-CNN-global	0.782/0.000	0.212
MVPD-CNN-hybrid	0.791/0.000	0.193

**Table 4:** Performance comparison of adaptive aesthetic model and MVPD-CNN-hybrid.

Method	Rp/Sig	MSE
MVPD-CNN-hybrid	0.791/0.000	0.193
IR_CNN_+SVR_DeepAesth_	0.823/0.000	0.161

## Data Availability

The data used to support this study are available from the corresponding author upon request.
